The article "A PCA-DEA-Based Model for Assessing the Sustainability of Marine Economy" was retracted in 2023. Reasons: unreliable results or conclusions; concerns about the data; concerns about the results or conclusions; concerns about the peer review.

# A PCA-DEA-Based Model for Assessing the Sustainability of Marine Economy

**DOI:** 10.1155/2022/2412588

**Published:** 2022-08-08

**Authors:** Haihui Yao, Jianping Huang, Junhua Li

**Affiliations:** ^1^School of Civil Engineering, Anyang Normal University, Anyang 455000, China; ^2^College of Chemistry and Chemical Engineering, Anyang Institute of Technology, Anyang 455099, China

## Abstract

One of the most important and continuously growing research areas in marine ecology is assessing the sustainability of ecosystems. The concept is traditionally approached by quantifying different anthropogenic pressures, such as top-down effects, overexploitation, invasive species, overfishing, and pollution. However, this perspective has been criticized for its inability to capture the complex interactions between natural factors (such as climate change), human factors, and sociopolitical factors that shape ecosystems. In this paper, we present a new structural model for assessing the sustainability of marine ecosystems, PCA-DEA-based model, as an extension to current models that incorporates these key interfaces into dynamic system modeling by including trade-offs on horizontal scales (e.g., decision making).

## 1. Introduction

The term “sustainability” has become a widely used concept in relation to the management and conservation of natural resources. The central aspect of sustainability is commonly considered to be maintenance of ecosystem services and social-ecological system (SES) functions over time. However, maintaining ecosystem services and SES functions requires managing the driving forces that affect them in a way that they do not collapse or become unsustainable.

The ideal situation would be to keep SES functions while limiting or even avoiding anthropogenic pressures (such as pollution and habitat destruction) that could threaten those functions. This, however, is quite a difficult task to achieve in the face of economic and sociopolitical pressures. Sustainability therefore depends on the interaction between different levels of scale and the decisions that we make at each level. In particular, it is crucial to pay attention to symbiotic relations between humans and nature that are embedded in complex social-ecological systems [1–3].

Human activities can have a profound impact on biodiversity, ecosystems, and SES functions [4]. We may be struggling against threats such as overfishing or pollution but also for reasons that are not necessarily anthropogenic. Climate change, for example, might emerge as a major threat to marine ecosystem sustainability over the coming years. In fact, researchers from the University of Victoria recently argued that climate change is one of the most important factors shaping marine ecosystems and that the effects are already observable (see http://marine-ecology.com/2013/03/13/climate-change-marine-ecosystems).

To support sustainable management decisions in this complex social-ecological system, we need models that are capable of simultaneously incorporating various drivers and their interactions into one system analysis framework. In this paper, we present a new approach for analyzing marine ecosystems and the sustainability of their SES functions. Unlike traditional models, this approach incorporates the major factor of decision making into the system process.

This new approach is based on a multi-criteria decision making (MCDM) framework that allows for an integrated assessment of sustainability issues and management strategies. In particular, we present a PCA-DEA-based model (PCA stands for Principal Components Analysis, and DEA stands for Dynamic Evolutionary Algorithm) that assesses the sustainability of marine economy. This model is an extension to current models that incorporates these key interfaces into dynamic system modeling by including trade-offs on horizontal scales [5–7].

The rest of the paper is structured as follows. We first give a brief introduction to the key concepts in MCDM and PCA-DEA modeling in Section 2.  Section 3 presents the model structure, and Section 4 illustrates the application of the model in a case study. We conclude with our main findings in Section 5.

### 1.1. MCDM Model

The basic idea behind MCDM analysis is to develop a comprehensive assessment of sustainability issues by simultaneously incorporating various drivers (e.g., fishing pressure, trawling) and their interactions into one model framework. The key inputs to MCDM are the relationships between key drivers (e.g., current fisheries intensity, trawling). However, these relationships are subject to change due to changes in human behaviour or even wildlife migration or through bottom-up impacts (bottom-up effects).

The model used in this paper is based on partial least square-discriminant analysis (PLS-DA) and differential evolution (DE). The model, however, is designed as a flexible tool that can be modified to fit a wide range of systems. It can be used to assess the impact of different drivers on different SES functions or evaluate critical points where trade-offs arise between two or more of them.

## 2. Method

The general idea behind the model is that it can be used to evaluate trade-offs between different components (such as SES functions or pressure) using a structural equation modeling (SEM) framework. SEM provides an effective tool for testing causal relationships among latent variables—that is, it allows for determining how much each of the latent variables affects the outcome variable. To do this, SEM typically consists of four stages specifying the conceptual model of a system to be modeled in terms of potential causality and correlation):

1. Defining nodes [8, 9] and variables that are used to measure them
2. Defining relations between variables (correlation)
3. Specifying the causal structure (chains)
4. Defining the functional form and estimating model parameters

The causal structure of the model is defined as a set of causal formulas and links between different variables that define which relations hold between them. In our case, each formula is a differential equation that links SES functions with pressure. The partial differential equations are stochastic in nature (that is, they are random), which increases their flexibility to fit multiple systems. The differential equations can be solved by a variety of methods such as particle filtering techniques [10]. However, it is more efficient to use an evolutionary algorithm that can solve thousands of equations in parallel [11].

### 2.1. Literature Review

Sustainability can be defined as the ability of a system to sustain its structure and functions [12]. Therefore, sustainability demands that we “balance” the management of ecosystems and their SES functions. Balancing however requires that we acquire deep insights into interactions between all major factors driving the system.

In this section, we review some of the major factors that drive marine ecosystems and discuss how they influence SES functions.

#### 2.1.1. Fishing Pressure

Fishing pressure is one of the major drivers that can have a profound impact on marine ecosystems. The results of fisheries research, in particular, suggest that overfishing and degraded ecosystem functions will continue to be major problems in the coming years [13].

However, fisheries are a very complex system. For example, fishing pressure can be direct or indirect and depends on legal frameworks related to anchoring or harvesting. Furthermore, it can have positive impacts on other functions such as ecotourism if managed properly. In order to properly evaluate the sustainability of marine economies we need to get better understanding of these underlying factors [14, 15] and their interactions.

#### 2.1.2. Marine Tourism

The recreational fishing industry plays a major role in the national economy of most countries (Lincoln and Shackelford, 2005). In fact, recreational fishing is responsible for approximately $48 billion USD to the US economy alone every year. However, this activity is dependent on marine ecosystems and their key SES functions [16]. In order to regulate this sector of the economy, we need to understand how different parameters such as tourism activities affect ecosystem functions [17].

#### 2.1.3. Trawling

Trawling is a particularly harmful form of fishing that has been devastating many marine ecosystems around the world [18]. The pressure exerted by trawling vessels is such that it can have a negative impact on key SES functions in some cases. However, together with other fishing methods, trawling can also be used as a management tool that can be used to maintain the health of certain SES functions [19]. Therefore, we need to understand which parameters drive the impacts of trawling.

### 2.2. Bottom-Up Effects

Bottom-up effects are also known as bottom-up pressures or heretofore undiscovered effects and are critical because they play an important role in driving the loss of ecosystems and their SES functions [20]. In a recent study, for example, it is shown that the loss of coral reefs can be driven by climate change and overfishing [21]. These complex interactions are difficult to detect as we rarely have complete information on different SES functions and their relationships.

The problem described above is potentially solvable if we use an integrative modeling approach that can combine many separate models into one framework. This framework can be used to address the following questions:

1. How much of each of the SES functions will remain under different fishing scenarios (e.g., sustainable fisheries)?
2. What are the critical points where ecosystem functions become unsustainable?
3. What are the major drivers that have a strong influence on the structure of the ecosystem and its SES functions?

The goal of this kind of framework is to provide better management solutions by allowing us to make better decisions. Therefore, it is important that we understand how marine ecosystems and their SES functions work in order to achieve sustainability.

In order to obtain some insight into these complex interactions, we will use an integrated modeling method that combines multiscale modeling with evolutionary algorithms. In the process, we will use a simple but effective differential equation model which can be solved using particle filtering methods [22].

## 3. Method

Research is conducted with a descriptive approach of mixed methods (quantitative-qualitative). The data used is secondary data obtained from statistical sources and scientific literature reviews. Data processing is carried out using linear regression analysis of the ordinary least square (OLS) method in the data period of 2011–2020. The mathematical model formed is as follows:

(1) $$\begin{array}{c} Y=\;\beta_{0}+\beta_{1}.\;X_{1}+\;\beta_{2}.\;X_{2}+\beta_{3}.\;X_{3}+\;\beta_{4}.\;D+\;\varepsilon , \end{array}$$

(2) $$\begin{array}{c} EG=\;C+\beta_{1}.\;G\;DP+\;\beta_{2}.\;TR+\beta_{3}.\;G+\;\beta_{4}.\;TA+\;\varepsilon \text{,} \end{array}$$

where EG is the economic growth (in percent); GDP is the gross domestic product (in billions of rupiah); TR is the tax revenues (in billions of rupiah); G is the government expenditures (in billions of rupiah); TA is the dummy variable of tax amnesty policy, divided by a binary number: 0 for period before implementation (2011–2015) and 1 for period after implementation (2016–2021).

After regression analysis of the model estimation, the next is residual testing through 3 classical assumption tests, namely, normality, multicollinearity, and autocorrelation. Normality tests are performed to see the residual distribution conditions of the data. The normality test is carried out by the Jarque–Bera method. If the *p* value is less than *α* (0.05), it means that residual data is not normally distributed. Multicollinearity tests are conducted with the aim of knowing the correlation between independent variables. Testing is done with the pairwise method. If the correlation value is above 0.8, it means that there is a multicollinearity problem in residual data. The autocorrelation test is conducted with the aim of knowing the existence of variable correlations in the prediction model with changes in time. Testing is conducted through the BG serial LM test. If the Prob. F value is less than *α* (0.05), it means that there is autocorrelation problem in the prediction model. Model estimation should be free from the problem of testing classical assumptions. If there is a problem, it is necessary to make improvements to the model.

## 4. Result and Discussion

### 4.1. Descriptive Analysis

Data on tax revenue statistics in Indonesia shows that in the last ten years the trend of tax revenues has tended to rise. In 2011, the tax revenue rate was Rp 878.685,22 billion. Until 2016, the rate of tax revenue has always increased. Growth in tax receipts from 2012 to 2016 was 15,65%, 13%, 8,51%, 19,51%, and 3,35%. In the period 2011 to 2021, the highest tax revenue rate occurred in 2015, which amounted to Rp 243.148,53 billion. Tax revenues also decreased in 2017 and 2020. The largest tax decrease occurred in 2020, which amounted to Rp 381.871,15 billion or equivalent to 21,38% compared to the previous year. Overall, in the last 11 years, tax revenues in Indonesia rose by Rp 525.822,28 billion or equivalent to 59,84%. If viewed in the period before and after the implementation of tax amnesty volume 1 of president Joko Widodo's leadership, which is in 2016, the average tax revenue per year was Rp 1.564.171,55 billion, while before the tax amnesty volume 1, the average tax revenue per year was Rp 1.155.729,94 billion; therefore, after the tax amnesty volume 1, it can be concluded that the average tax revenue per year is greater than Rp 408.441,61 billion when compared to the period before enactment of tax amnesty volume 1 as shown in Table 1.

Almost the same as the trend of tax revenues, data on the gross domestic product (GDP) rate also has a trend that tends to rise in the last 11 years. The GDP data shown is the GDP spending approach based on constant price of 2010 base year. In 2011, Indonesia's GDP amounted to Rp 7.287.635,3 billion. The following year, GDP increased by Rp 439.448,1 billion. Overall, the largest GDP increase occurred in 2019, amounting to Rp 523.185,9 billion. But in the following year, GDP actually decreased quite sharply, amounting to Rp 226.595,1 billion. This happened because of the COVID-19 pandemic that made the activities of almost all sectors of economy difficult to run. Economic growth data that is a reflection of the increase in GDP automatically also has the same trend as GDP. The largest increase in economic growth occurred in 2016, which was 0,15 basis points compared to the previous year. As for the largest decline in economic growth occurred in 2020, which amounted to 7,09 basis points compared to 2019. The average economic growth per year after tax amnesty volume 1 is 3,64%. This figure is smaller than that before enactment of tax amnesty volume 1. This indicates a slowdown in economic growth in the last 5 years as shown in Table 2.

Government expenditures as one of the constituent components of GDP must also be analyzed for its development. The increase in government expenditures from 2011 to 2021 has a trend tending to rise. In 2011 government expenditure was at Rp 1.320.752,32 billion. Then, it increased by Rp 227.559,02 billion, equivalent to 17,23%, the following year. The largest increase in government expenditures occurred in 2012, while the smallest increase in government expenditures occurred in 2017, amounting to Rp 50.347,02 billion or equivalent to 2,42% compared to the previous year. The average government expenditures before the enactment of tax amnesty volume 1 are Rp 1.691.255,09 billion per year. Meanwhile, since 2016, the average government expenditure has risen to Rp 2.327.435,94 billion per year. This can be interpreted by the fact that, in the last 5 years, the government has been more active in doing shopping. Overall, in the last 11 years, there has been an increase in government expenditures of Rp 1.418.414,55 billion or equivalent to 107,39% when compared to the figure in 2011.

### 4.2. Empirical Analysis

As shown in Table 3, from the results of the data processing using ordinary least square regression, all variables have been in order with the theory. From the results of the estimated output, the mathematical model can be written as follows:

(3) $$\begin{array}{c} EG=2,47+3,80\;LOG\left(GDP\right)+1,36\;LOG\left(TR\right)+2,52\;LOG\;\left(G\right)+0,07\;TA+\;\varepsilon . \end{array}$$

Judging from the coefficient value, all independent variables have a positive effect on dependent variables. As a proof of the validity of empirical evidence, it has been tested on data, starting from residual testing through classical assumption tests and then testing data as proof of hypothesis and interpretation of coefficient of determination.

#### 4.2.1. Classical Assumption Test

The normality test is performed to test the residual results of the model estimate. Three types of residual testing were done, namely, normality test, multicollinearity test, and autocorrelation test. This is done based on consideration of the data used. Normality test was conducted using the Jarque–Bera (JB) method. The resulting *p* value is at 0.5984. From these results, it can be concluded that the *p* value > 0.05. This means that residual data is normally distributed as shown in Figure 1.

Multicollinearity problem detection was done through pairwise correlation testing. Multicollinearity test results showed that the correlation coefficient of all variables was less than 0.8. This means that there is no multicollinearity problem in the model tested as shown in Table 4.

Next is the detection of autocorrelation problems done through LM test. From the test, we obtained the result that the value of Prob. F amounted to 0.5251. This means that Prob.* *F value > 0.05, so it can be concluded that there are no autocorrelation problems in the model as shown in Table 5.

#### 4.2.2. Hypothesis Testing

Hypothesis testing is done with two approaches: partial and simultaneous. Partial tests are conducted through a comparison of *t* table and *t* statistics, while the simultaneous test is conducted through the comparison of F table value and F statistics value as shown in Table 6.

From the results of partial tests through comparisons of *t* tables and *t* statistics, all independent variables have a statistical *t* value greater than *t* tables, meaning that the variables gross domestic product, tax revenues, government expenditures, and tax amnesty each have a significant effect on the variable economic growth. Partial tests can also be performed by looking at the Prob. value of each variable. If the Prob. value < 0.05, it means that the variable has a significant influence as shown in Table 7.

Simultaneous hypothesis testing conducted through the comparison of F tables and statistical *F* shows that F statistics > *F* tables, meaning that simultaneously all independent variables have a significant effect on dependent variables.

#### 4.2.3. Determination Coefficient

The regression results through ordinary least square show that the value of R-squared is 0.9325. This means that all independent variables are able to explain the state of independent variables by 93,25% as shown in Table 8.

### 4.3. Coefficient Interpretation

From the coefficient value of the data processing, we can see the magnitude of the influence of each variable. The constant coefficient is 2.47. This means that when all independent variables do not change, the economy will continue to experience growth of 2,47%. This is thought to occur because the presence of other variables (beyond the variables studied) affects the economic sector. The LOG (GDP) variable has a coefficient of 3.80 meaning that when GDP rises by 1%, the economy will grow by 3,8%. The tax revenues variable has a coefficient of 1.36. This means that when tax revenues rise by 1%, the economy will grow by 1,36%. Furthermore, the government expenditures variable has a coefficient of 2.52. This means that when government spending rises by 1%, the economy will grow by 2,52%. Then, the dummy variable tax amnesty also shows a significant positive influence, which is at a coefficient of 0.07. This means that there is a difference in economic growth of 0,07% after the tax amnesty policy volume 1.

## 5. Discussion

In general, economic growth figures in Indonesia have been outlined in the “Descriptive Analysis.” The value of economic growth discussed is economic growth in general. In the period 2011–2021, it is seen that the average economic growth before tax amnesty is actually slightly higher than that after tax amnesty volume 1. However, this cannot be fully attributed to the taxation aspect, considering that economic growth in Indonesia is influenced by many factors. In the current COVID-19 pandemic conditions, economic conditions in previous times will feel biased if used as a benchmark, considering the cause of the current recession is difficult to predict when it ends. The government's efforts to re-implement the tax amnesty policy to speed up economic recovery are a step worth considering. Compared to other countries, the implementation of the tax amnesty in Indonesia is arguably a success. The declared price value reached 39.5% of gross domestic product (GDP), far above countries such as India, Spain, or Italy which previously also implemented a tax amnesty. Meanwhile, the Rp 14.23 trillion ransom was equivalent to 1.08% of GDP at that time, higher than similar programs in Germany, Belgium, and Australia. Several efforts have been made to encourage economic growth and reduce poverty; one of them is achieved through increasing government spending. Government expenditure is part of fiscal policy, namely, an action by the government to regulate the course of the economy through budget. Government spending is needed to increase physical capital such as infrastructure basic and public facilities, as well as for the improvement of public services such as health, education, social protection, order and peace, and the environment, which in turn can improve the economy and social welfare. One of the targets of government spending is to increase production capacity and maintain sustainable growth economy. In realizing this goal, government spending is usually allocated to fixing infrastructure because all economic activities require adequate facilities and infrastructure. The effectiveness of government spending on development performance in Indonesia has been widely studied by researchers. Abdullah and Rusdarti's study (2017) reveals that government spending in developing countries such as Indonesia, Malaysia, Singapore, Ethiopia, Nigeria, and India and developed countries in Europe have positive influence on economic growth.

### 5.1. Projection of Re-implementation of Tax Amnesty Policy

The reintroduction of tax amnesty is a chance for taxpayers to reveal tax liabilities that have not been paid voluntarily by paying income tax based on asset disclosure. Many advantages will result from the adoption of this policy, including the removal of administrative punishments for taxpayers and data protection in the form of the revealed property data not being used as a basis for inquiry, investigation, or criminal prosecution of taxpayers.

If those advantages are linked to economic development, then the re-implementation of the tax amnesty is expected to boost economic growth. Starting with the rising number of assets raised, there will be a lot of ransom, which will result in a rise in tax revenues. The budgetary foundations of the government are strengthened by greater tax receipts. The government's ability to spend money is increasing. The economic environment will improve, resulting in more economic activity, lower unemployment, and higher economic growth. However, as stated in the “Introduction” and “Literature Review,” adopting this policy necessitates a number of difficult considerations in order to fulfill the goals established.

### 5.2. Implication

The study's findings suggest that tax amnesty has been experimentally proved to boost economic development in a favorable manner. However, when compared to other factors, its impact on economic development seems to be the least. The government must evaluate the level of GDP and government expenditures if the goal is to boost economic growth. When considering a tax amnesty scheme, the state of political stability must also be taken into account. Furthermore, the procurement of tax amnesty does not have to avoid long-term length and frequency too often since it is believed that it would alter taxpayer behavior. This lends credence to Ibrahim's study (2017).

## 6. Conclusion

Because taxes are the primary source of governmental revenue, their movement is critical. The situation of economic circumstances that have slowed since 2018 is worth considering. Tax amnesty is an issue worth addressing in analyzing economic development, given the amount of studies that show it may enhance tax compliance while failing to fulfill tax revenue objectives. Taxes are components that impact a country's disposable income, which is expressed in the form of GDP. Government spending, which includes both central government spending and monies distributed to the area, is also a factor in determining the pace of economic growth, particularly when using the GDP spending method. The findings of time series data regressed OLS revealed that GDP, tax revenues, government expenditures, and tax amnesty all had a substantial influence on economic growth, partly and concurrently. The findings also revealed that the pace of economic development differed before and after the introduction of tax amnesty volume 1 in 2016. Tax amnesty is a good way to stimulate economic development, but it must take into consideration political circumstances, length, and frequency of implementation. Only yearly data from 11 periods and four independent variables were included in the research. Further study is intended to employ data with more specific frequencies in order to better define the policy implementation cut-off point. The variables utilized are macroeconomic indicators in general; however, further study may be done to add or replace variables with indicators that are more relevant to tax theory.

## Figures and Tables

**Figure 1:** Output of normality test.

**Table 1:** Tax revenue and gross domestic product of Indonesia on 2011–2021.

Year	Tax revenues (billions of rupiah)	GDP (billions of rupiah)
**2011**	878.685,22	7.287.635,30
**2012**	1.016.237,34	7.727.083,40
**2013**	1.148.364,68	8.156.497,80
**2014**	1.246.106,96	8.564.866,60
**2015**	1.489.255,49	8.982.517,10
**2016**	1.539.166,24	9.434.613,40
**2017**	1.472.709,86	9.912.928,10
**2018**	1.618.095,49	10.425.851,90
**2019**	1.786.378,65	10.949.037,80
**2020**	1.404.507,50	10.722.442,70
**2021**	1.444.500,30	11.118.868,50

Source: Indonesian Central Bureau of Statistics, 2022.

**Table 2:** Government expenditure and GDP growth of Indonesia in 2011–2021.

Year	Government expenditures (billions of rupiah)	GDP growth (%)
**2011**	1.320.751,32	6.17
**2012**	1.548.310,34	6.03
**2013**	1.726.191,30	5.56
**2014**	1.876.872,76	5.01
**2015**	1.984.149,71	4.88
**2016**	2.082.948,90	5.03
**2017**	2.133.295,92	5.07
**2018**	2.220.656,97	5.17
**2019**	2.461.112,04	5.02
**2020**	2.739.165,87	−2.07
**2021**	2.786.809,38	3.69

Source: Indonesian Central Bureau of Statistics, 2022.

**Table 3:** Output of multiple regression.

Variable	Coefficient	Std. error	*t* statistic	Prob.
*C*	2.475245	1.039703	2.380722	0.0037
LOG (GDP)	3.802031	1.418237	2.680815	0.0262
LOG (TR)	1.365366	0.338075	4.038644	0.0099
LOG (*G*)	2.520684	0.592713	4.252785	0.0081
TA	0.074447	0.032145	2.315960	0.0376
R-squared	0.932529			
F-statistic	17.27660			
Prob. (F-statistic)	0.003939			

Source: data processed, 2021.

**Table 4:** Output of multicollinearity test.

	LOG (GDP)	LOG (TR)	LOG (G)	TA
LOG (GDP)	1.000000	0.516321	0.567335	0.576089
LOG (TR)	0.516321	1.000000	0.575004	0.548830
LOG (G)	0.567335	0.575004	1.000000	0.591450
TA	0.576089	0.548830	0.591450	1.000000

Source: data processed, 2021.

**Table 5:** Output of autocorrelation test.

Breusch–Godfrey serial correlation LM test			
F-statistic	0.804639	Prob. F (2, 3)	0.5251
Obs^*∗*^R-squared	3.491389	Prob. Chi-Square (2)	0.1745

Source: data processed, 2021.

**Table 6:** Output of partial hypothesis testing.

Variable	Df	*t* table	Abs *t* stat	Result
LOG (GDP)	9	2,26	2,68	H_0_ rejected, H_a_ accepted
LOG (TR)	9	2,26	4,03	H_0_ rejected, H_a_ accepted
LOG (G)	9	2,26	4,25	H_0_ rejected, H_a_ accepted
TA	9	2,26	2,31	H_0_ rejected, H_a_ accepted

Source: data processed, 2021.

**Table 7:** Results of simultaneous hypothesis testing.

Variable	Df1	Df2	F table	Abs F stat	Result
All variables	5	4	6,26	17,27	H_0_ rejected
					H_a_ accepted

Source: data processed, 2021.

**Table 8:** Determination coefficient.

R-squared	0.932529	Mean dependent var	4.587000

Adjusted R-squared	0.878553	Std. dev. dependent var	2.382161

Source: data processed, 2021.

## Data Availability

The data used to support the findings of this study are included within the article.

## Additional Points

*Limitations*. The authors acknowledge that there are certain limitations to their research. This research solely looked at economic circumstances for 11 years and only focused on tax amnesty policy volume 1 during the working cabinet period (during President Joko Widodo's presidency), even though comparable policies had been implemented earlier. The condition of economic development following the relaxing of PPKM was also overlooked in this research. Other factors are ignored in this analysis, which focuses only on fiscal variables. General economic growth is used as the dependent variable. Further study is required to address the identified flaws in order to provide more relevant policy suggestions.
